The article "Survival analysis of comprehensive treatment in Chinese patients with metastatic melanoma: A retrospective analysis" was published in 2024. Journal: Skin Res Technol.

# Survival analysis of comprehensive treatment in Chinese patients with metastatic melanoma: A retrospective analysis

**DOI:** 10.1111/srt.13546

**Published:** 2024-01-26

**Authors:** Qianqi Chen, Yan Zhao, Pupu Li, Jiangman Duan, Xiaohong Fu, Yueqiang Tang, Yinan Ma, Qiming Zhou

**Affiliations:** ^1^ Department of Internal Medicines, Oncology Huazhong University of Science and Technology Union Shenzhen Hospital Shenzhen Guangdong Province PR China

**Keywords:** immune checkpoint inhibitors (ICIs), malignant melanoma, PD‐1 mAb, survival analysis

## Abstract

**Background:**

Most of the current progression of immune checkpoint inhibitors for malignant melanoma is based on data from Caucasians in Western countries, but the benefit of Chinese patients is limited, mainly due to different pathological subtypes. The patients in western countries are mainly skin melanoma (about 90%), while the acral and mucosal types are dominant in China, accounting for 41.8% and 22.6% respectively. Acral and mucosal melanoma have lower response rates to immunotherapy and chemotherapy.

**Objective:**

Whether immune checkpoint inhibitors can improve the survival of Chinese patients with malignant melanoma, therefore, we conducted a retrospective analysis.

**Methods:**

We analyzed 53 patients with metastatic melanoma treated in our hospital to evaluate the efficacy and safety of PD‐1 mAb in Chinese patients with metastatic melanoma, and performed univariate and multivariate analyses of prognostic factors that may affect overall survival (OS).

**Results:**

In a study of 125 patients with advanced malignant melanoma, 53 patients participated, with a median follow‐up of 16 months. Among these, 69.8% died, and 30.2% remained on treatment. Median progression‐free survival (PFS) was 6 months, and median OS was 19 months. Patients treated with immune checkpoint inhibitors had improved outcomes, with a median PFS of 7 months and a median OS of 24 months. Patients with bone metastasis and aberrant Lactate dehydrogenase (LDH) post‐treatment had worse prognoses, while immunotherapy was a protective factor. Subgroup analysis showed the benefits of immunotherapy across various patient characteristics. No unexpected toxicities were observed.

**Conclusion:**

The study highlights the efficacy of immune checkpoint inhibitors, particularly PD‐1 mAb, in improving survival outcomes for Chinese patients with metastatic melanoma.

## 1 INTRODUCTION

Currently, immune checkpoint inhibitors (ICI) have greatly improved the prognosis of advanced malignant melanoma. Immune checkpoint inhibitors, such as Ipilimumab, nivolumab, and pembrolizumab, have been successively approved by the US Food and Drug Administration for the treatment of advanced metastatic melanoma.^1^, ^2^ Most of the current progression of immune checkpoint inhibitors for malignant melanoma is based on data from Caucasians in Western countries, but the benefit of Chinese patients is limited, mainly due to different pathological subtypes. The patients in western countries are mainly skin melanoma (about 90%), while the acral and mucosa types are dominant in China, accounting for 41.8% and 22.6% respectively.^3^, ^4^, ^5^ Compared to cutaneous malignant melanoma, acral and mucosal melanomas are generally considered more aggressive malignancies, exhibiting low response rates to immunotherapy and chemotherapy.^6^, ^7^, ^8^ In a retrospective analysis, the objective response rate (ORR) of ipilimumab, pembrolizumab and pembrolizumab plus ipilimumab were 0%, 25% and 20%, respectively.^9^ In the KEYNOTE‐151 study, the objective response rates in mucosal and acral melanoma of Chinese advanced melanoma patients were 13.3% for pembrolizumab and 15.8% (ORR),^10^ respectively, median progression‐free survival (PFS) 2.8 months, and median overall survival (OS) 12.1 months.^11^ Poor options for advanced malignant melanoma in China. Before 2017, the first‐line treatment of advanced melanoma in China was dominated by dacarbazine‐based chemotherapy. The median survival time of chemotherapy for patients with advanced melanoma is 6–9 months, with a 5‐year survival rate of less than 10%^12^.

The article "Survival analysis of comprehensive treatment in Chinese patients with metastatic melanoma: A retrospective analysis" was published in 2024. Journal: Skin Res Technol.

To determine whether immune checkpoint inhibitors can enhance the survival of Chinese patients with malignant melanoma, we conducted a retrospective analysis of 53 patients with metastatic melanoma treated at our hospital. This study aimed to assess the efficacy and safety of PD‐1 mAb in Chinese patients with metastatic melanoma and perform univariate and multivariate analyses of potential prognostic factors impacting OS.

## 2 MATERIALS AND METHODS

### 2.1 Patient population

We included patients aged at least 18 years, we enrolled patients who were at least 18 years of age, with pathologically confirmed locally advanced or metastatic melanoma. Patients met the following inclusion criteria: (1) Patients must have at least one measurable lesion at baseline according to the Response Assessment criteria for solid tumors (RECIST version 1.1). (2) The Eastern Cooperative Oncology Group (ECOG) fitness status of 0 or 1, with adequate organ and bone marrow function. (3) Patients with an expected survival period of more than 3 months. (4) Patients who have received at least 1 cycle of first‐line anti‐tumor therapy before December 31, 2021. (5) Patients receiving full drug treatment in our department. Patients with an autoimmune disease were excluded.

The article "Survival analysis of comprehensive treatment in Chinese patients with metastatic melanoma: A retrospective analysis" was published in 2024. Journal: Skin Res Technol.

### 2.2 Study design and follow‐up

This study is a retrospective cohort study. Patients with locally advanced or metastatic malignant black melanoma treated in our department, were divided into immunotherapy group and non‐immunotherapy groups. Patient's clinical characteristics, treatment regimen, treatment lines, efficacy assessment, adverse reactions, disease progression, cause of death, were tracked and recorded until October 31, 2022 or until the death of the patient. Patients eligible for enrollment in this study, underwent a survival analysis.

### 2.3 Statistical analysis

PFS and OS were plotted using the Kaplan‐Meier method, reporting the median and corresponding two‐sided 95% CI, with a *p*‐value < 0.05 considered statistically significant. PFS was defined as the time from PD‐1, onset to disease progression or death (whichever comes first) as determined by RECIST 1.1. OS was defined as the time from the start of first‐line treatment to death from any cause. The log‐rank test was used to compare the correlation between baseline characteristics and OS. A Cox proportional hazards regression analysis was used to determine the relative impact of the identified prognostic factors. The multiple cox regression analysis was performed using reverse stepwise (LR) for variables with *p*‐value < 0.1 in univariate cox regression analysis. In the multivariate cox regression analysis, variables with a *p*‐value < 0.05 were considered as independent prognostic factors for melanoma patients.

## 3 RESULTS

### 3.1 Patients and treatment

From January 1, 2015 to December 31, 2021, 125 patients with advanced malignant melanoma were screened in Department of Internal Medicines, Oncology, Huazhong University of Science and Technology Union Shenzhen Hospital, and 53 patients participated in the study. The median age was 49.5 years (range 18–86), with 19 (35.8%) male patients and 34 (64.2%) female patients. Among the melanoma subtypes, 10 (18.9%) were cutaneous malignant melanomas, 26 (49.1%) were acral malignant melanomas, and 17 (32.1%) were mucosal malignant melanomas, which is roughly in proportion to the current pathological classification of malignant melanoma in China. Thirteen (24.5%) patients were tested for the BRAF V600E mutation and 6 (11.3%) patients were tested for MDM 2 amplification. The common metastatic sites in the late stage of initial diagnosis include lymph nodes (92.5%), lung (49.1%), bone (24.5%), subcutaneous tissue (18.9%), liver (17%), brain (17%), and so forth. The majority of patients (96.2%) had a ECOG PS score of 1. LDH levels increased by 32.1%. More than half (67.9%) of the patients had received at least two or more lines of treatment. Forty‐three (81.1%) had received immune checkpoint inhibitors, 41 (77.4%) had received systemic chemotherapy, 37 (69.8%) had received targeted drugs, and 33 (62.3%) had received topical therapy. Baseline characteristics are shown in Table 1.

The article "Survival analysis of comprehensive treatment in Chinese patients with metastatic melanoma: A retrospective analysis" was published in 2024. Journal: Skin Res Technol.

**TABLE 1:** Demographics of study participants.

Characteristic	*N* (%)
**Gender**	
Female	34 (64.2)
Male	19 (35.8)
**Age**	
<60y	37 (69.8)
≥60y	16 (30.2)
**Histology**	
Skin	10 (18.9)
Acral	26 (49.1)
mucosal	17 (32.1)
**Clark grade**	
0	29 (54.7)
1	3 (5.7)
2	1 (1.9)
3	2 (3.8)
4	8 (15.1)
5	10 (18.9)
**ECOG PS**	
0–1	51 (96.2)
2	2 (3.8)
**LDH**	
Normal	36 (67.9)
Abnormal	17 (32.1)
**Lung MET**	
No	27 (50.9)
Lung MET	26 (49.1)
**Liver MET**	
No	44 (83.0)
Liver MET	9 (17.0)
**Brain MET**	
No	44 (83.0)
Brain MET	9 (17.0)
**Bone MET**	
No	40 (75.5)
Bone MET	13 (24.5)
**LN MET**	
No	4 (7.5)
LN MET	49 (92.5)
**Skin MET**	
No	43 (81.1)
Skin MET	10 (18.9)
**BRAF**	
Wild type	32 (60.4)
Mutant type	13 (24.5)
Not available	8 (15.1)
**CKIT**	
Wild type	26 (49.1)
Mutant type	2 (3.8)
Not available	25 (47.2)
**NRAS**	
Wild type	28 (52.8)
Mutant type	2 (3.8)
Not available	23 (43.4)
**MDM2**	
Negative	33 (62.3)
Amplification	6 (11.3)
Not available	14 (26.4)
IO status	
IO	43 (81.1)
No	10 (18.9)
**Chemo**	
Yes	41 (77.4)
No	12 (22.6)
**Targeted**	
Yes	37 (69.8)
No	16 (30.2)
**Local**	
Yes	33 (62.3)
No	20 (37.7)

Abbreviations: IO, immuno‐oncology, HR, hazard ratio, ECOG, eastern cooperative oncology group; LDH, lactate, dehydrogenase, MET, metastasis, LN MET, lymph node metastasis, CKIT, a gene encoding the receptor tyrosine kinase protein known as tyrosine‐protein kinase KIT, also known as CD117, NRAS, neuroblastoma RAS viral oncogene, that encodes an enzyme also called as NRAS enzyme, and MDM2, a gene that encodes a protein called as mouse double minute 2 homolog (MDM2).

Immune checkpoint inhibitor therapy in this study included PD‐1 (Pembrolizumab, Nivolumab, and Toripalimab) and CTLA‐4 (Ipilimumab). Chemotherapeutic drugs include albumin paclitaxel, temozolomide, dacarbazine and cisplatin, and so forth. Targeted drugs include BRAF inhibitors (dabrafenib, Vemurafenib), MEK inhibitors (Trametinib), and antiangiogenic agents (Bevacizumab, Lenvatinib). Forty‐three patients were treated with immune checkpoint inhibitors, as compared with 10 patients (Table 2). Twelve patients in the immunotherapy group were on BRAF inhibitor and one patient in the no immunotherapy group was on BRAF inhibitor. More than half of the patients who had not been treated with immune checkpoint inhibitors did not undergo genetic testing.

**TABLE 2:** Patients characteristics comparison between patients with or without IO.

	IO 43 (%)	Without IO 10 (%)	*p*‐value
**Gender**			0.092
Female	28 (65.1)	6 (60.0)	
Male	15 (34.9)	4 (40.0)	
**Age**			0.050
<60 years	33 (76.7)	4 (40.0)	
≥60 years	10 (23.3)	6 (60.0)	
**Histology**			0.638
Skin	9 (20.9)	1 (10.0)	
Acral	20 (46.5)	6 (60.0)	
Mucosal	14 (32.6)	3 (30.0)	
**Clark**			0.725
0–2	26 (60.5)	7 (70.0)	
3–5	17 (39.5)	3 (30.0)	
**ECOG PS**			1.000
0–1	41 (95.3)	10 (100.0)	
2	2 (4.7)	0 (0.0)	
**LDH**			0.058
Normal	32 (74.4)	4 (40.0)	
Abnormal	11 (25.6)	6 (60.0)	
**Lung MET**			0.293
No	20 (46.5)	7 (70.0)	
Lung MET	23 (53.5)	3 (30.0)	
**Liver MET**			0.346
No	37 (86.0)	7 (70.0)	
Liver MET	6 (14.0)	3 (30.0)	
**Brain MET**			0.346
No	37 (86.0)	7 (70.0)	
Brain MET	6 (7.3)	3 (30.3)	
**Bone MET**			1.000
No	32 (74.4)	8 (80.0)	
Bone MET	11 (25.6)	2 (20.0)	
**LN MET**			1.000
No	4 (9.3)	0 (0.0)	
LN MET	39 (90.7)	10 (100.0)	
**Skin MET**			0.665
No	34 (79.1)	9 (90.0)	
Skin MET	9 (20.9)	1 (10.0)	
**BRAF**			0.007
Wild type	29 (67.4)	3 (30.0)	
Mutant type	12 (27.9)	1 (10.0)	
NA	2 (4.7)	6 (60.0)	
**CKIT**			0.213
Wild type	23 (53.5)	3 (30.0)	
Mutant type	2 (4.7)	0 (0.0)	
NA	18 (41.9)	7 (70.0)	
**NRAS**			0.135
Wild type	25 (58.1)	3 (30.0)	
Mutant type	2 (4.7)	0 (0.0)	
NA	16 (37.2)	7 (70.0)	
**MDM2**			0.003
Negative	31 (72.1)	2 (20.0)	
Amplification	5 (11.6)	1 (10.0)	
NA	7 (16.3)	7 (70.0)	
**Chemo**			0.423
Yes	32 (74.4)	9 (90.0)	
No	11 (25.6)	1 (10.0)	
**Targeted**			0.462
Yes	31 (72.1)	6 (60.0)	
No	12 (27.9)	4 (40.0)	
**Local**			0.112
Yes	29 (67.4)	4 (40.0)	
No	14 (32.6)	6 (60.0)	

Abbreviations: IO, immuno‐oncology, HR, hazard ratio, ECOG, eastern cooperative oncology group; LDH, lactate dehydrogenase, MET, metastasis, LN MET, lymph node metastasis, CKIT, a gene encoding the receptor tyrosine kinase protein known as tyrosine‐protein kinase KIT, also known as CD117, NRAS, neuroblastoma RAS viral oncogene, that encodes an enzyme also called as NRAS enzyme, and MDM2, a gene that encodes a protein called as mouse double minute 2 homolog (MDM2); BRAF, a human gene that encodes a protein called B‐Raf, while the protein is more formally known as serine/threonine‐protein kinase B‐Raf.

The article "Survival analysis of comprehensive treatment in Chinese patients with metastatic melanoma: A retrospective analysis" was published in 2024. Journal: Skin Res Technol.

### 3.2 Treatment‐related toxicity

Of the 43 patients receiving immunotherapy, 21 had immune‐related adverse effects, mostly grade 1–2, most commonly rash (8), hepatic insufficiency (5), and hypothyroidism (4). No other patients discontinued treatment due to immune‐related adverse reactions, and no other new adverse reactions were observed.

### 3.3 Antitumor activity

The median follow‐up time at the data cutoff (October 31, 2022) was 16.0 months (95% CI 7.848–24.152). In the intent‐to‐treat (ITT) population (*n* = 53), 37 (69.8%) died and 16 (30.2%) remained on treatment. Median PFS was 6 months and median OS was 19 months. For those patients treated with immune checkpoint inhibitors, the median PFS was 7 months, and the median PFS was 4 months without immunotherapy (*p* = 0.253, Table 3, Figure 1A). Patients receiving immune checkpoint inhibitors had a median OS of 24 months, and the median OS was 7 months (*p* = 0.001, Table 4, Figure 1B). Four (9.3%) of the patients receiving immune checkpoint inhibitors were still receiving PD‐1 as of the time of publication.

**TABLE 3:** Progression free survival comparison between patients with or without IO (date from first line to date of PD).

	Median	95% CI	*p*‐value
IO	7.000	5.188–8.812	0.253
Without IO	4.000	0.901–7.099	
Total	6.000	4.575–7.425	

Abbreviations: IO, immuno‐oncology.

**FIGURE 1:** Progression‐free survival and OS. Kaplan‐Meier survival curves for progression‐free survival between patients with or without IO (A) and overall survival (B) between patients with or without IO. OS, overall survival.

**TABLE 4:** Overall survival comparison between patients with or without IO (date from first line to date of events).

	Median	95% CI	*p*‐value
IO	24	17.028–30.972	0.001
Without IO	7	3.907–10.099	
Total	19	10.035–27.965	

Abbreviation: IO, immuno‐oncology.

Immune checkpoint inhibitor therapy included Pembrolizumab (69.8%), Toripalimab (16.3%), Pembrolizumab + Ipilimumab (9.3%), Nivolumab (2.3%), and so forth. Thirty (69.8%) patients were on first‐line treatment. Most of them were combination therapies, including immunocombination chemotherapy (41.9%) and targeted drugs (39.5%). Four patients (9.3%) had had the best efficacy of immunotherapy in CR, and 15 patients (34.9%) had achieved PR (Table 5).

**TABLE 5:** Data of patients who received IO therapy.

	Frequency (%)
**Line**	
Adjuvant	2 (4.7)
First line	30 (69.8)
Second line	10 (23.3)
Multiple line	1 (2.3)
**IO agent**	
Pembro	30 (69.8)
Nivo	1 (2.3)
Terriprizumab	7 (16.3)
Pembro+CTLA4	4 (9.3)
Others	1 (2.3)
**Treatment strategy**	
IO monotherapy	8 (18.6)
IO + chemo	18 (41.9)
IO + T argeted	17 (39.5)
**Best response of IO**	
CR	4 (9.3)
PR	15 (34.9)
SD	19 (44.2)
PD	3 (7.0)
NA	2 (4.7)
**PFS**	
Median (95% CI)	7.0 (5.035–8.695)
**OS**	
Median (95% CI)	23.0 (14.961–31.039)

Abbreviations: IO, immuno‐oncology, OS, overall survival; PFS, progression‐free survival.

This study also found that combined topical therapy showed a trend of survival benefit compared with no topical treatment. Local treatment included radiotherapy (23.43%), arterial perfusion therapy (16.30%), and ablation (7.13%). The median OS was 24 months versus 11 months for patients not (*p* = 0.327), as shown in Table 6.

**TABLE 6:** Overall survival comparison between patients with or without localized therapy (date from first line to date of events).

	Median	95% CI	*p*‐value
Localized	24.0	15.936–32.064	0.327
Without localized	11.0	4.459–17.541	
Total	19.0	10.035–27.965	

The article "Survival analysis of comprehensive treatment in Chinese patients with metastatic melanoma: A retrospective analysis" was published in 2024. Journal: Skin Res Technol.

### 3.4 Prognostic factors for melanoma patients

The results of univariate analysis showed that age 60 years (*p* = 0.029,95% CI: 1.079–3.983), high LDH (*p* = 0.001, 95% CI: 1.530–5.979), bone metastasis (*p* = 0.017, 95% CI: 1.167–4.971), immunotherapy (*p* = 0.002, 95% CI: 0.152–0.663),and chemotherapy (*p* = 0.032, 95% CI: 0.158–0.920) were related to OS (*p* < 0.1, Table 7). Variables with a *p* value < 0.1 in univariant COX‐regression analysis were selected for multivariant COX‐regression analysis by the Backward Stepwise (LR). Variables with a *p* value < 0.05 in multivariant COX‐regression analysis were considered as independent prognostic factors for melanoma patients. In this study, bone metastasis (*p* = 0.013, 95% CI: 1.057–4.606), aberrant LDH (*p* = 0.013, 95% CI: 1.211–5.007) post treatment were poor prognostic factors, while patients with IO therapy (*p* = 0.001, 95% CI: 0.113–0.545) were considered as protective factor for prognosis (Table 8).

**TABLE 7:** Univariant analysis of OS.

	*p*‐value	HR	95% CI
**Gender**			
Male/female	0.382	1.335	0.698–2.553
**Age**			
≥60 years/<60	0.029	2.073	1.079–3.983
**Histology**	0.528		
Acral/skin	0.730	1.168	0.484–2.821
Mucosal/skin	0.310	1.598	0.647–3.949
**Clark**			
3–5/0–2	0.435	0.769	0.398–1.486
**ECOG PS**			
2/0–1	0.429	1.785	0.424–7.520
**LDH**			
abnormal/normal	0.001	3.025	1.530–5.979
**Lung MET**			
MET/no	0.773	0.911	0.483–1.716
**Liver MET**			
MET/no	0.599	1.247	0.548–2.839
**Brain MET**			
MET/no	0.312	1.528	0.671–3.479
**Bone MET**			
MET/no	0.017	2.049	1.167–4.971
**LN MET**			
MET/no	0.427	1.783	0.4297.420
**Skin MET**			
MET/no	0.827	1.091	0.501–2.378
**BRAF V600E**	0.003		
Mutant/wild	0.341	0.675	0.300–1.517
NA/wild	0.003	3.726	1.562–8.886
**NRAS**	0.684		
Mutant/wild	0.980	0.0	0.0
NA/wild	0.384	1.325	0.704–2.494
**IO**			
IO/without IO	0.002	0.318	0.152–0.663
**Chemo**			
No/yes	0.032	0.381	0.158–0.920
**Targeted**			
No/yes	0.255	0.645	0.303–1.37
**Local**			
No/yes	0.337	1.384	0.713–2.687

Abbreviations: ECOG, eastern cooperative oncology group; LDH, lactate dehydrogenase, IO, immuno‐oncology,.

**TABLE 8:** Multivariate analysis of OS.

	*p*‐value	HR	95% CI
**Age**			
≥60 years/<60	0.192	1.684	0.107–1.326
**LDH**			
abnormal/normal	0.013	2.462	1.211–5.007
**Bone MET**			
MET/no	0.035	2.206	1.057–4.606
**BRAF**	0.317		
Mutant/wild	0.348	1.755	0.542–5.684
NA/wild	0.191	2.141	0.685–6.694
**IO**			
IO/without IO	0.001	0.248	0.113–0.545
**Chemo**			
No/yes	0.080	0.436	0.172–1.105

Abbreviations: LDH, lactate dehydrogenase, IO, Immuno‐oncology

Variables with a *p* value < 0.1 in univariant COX‐regression analysis were selected for multivariant COX‐regression analysis by the Backward Stepwise (LR). Variables with a *p*‐value < 0.05 in multivariant COX‐regression analysis were considered as independent prognostic factors for melanoma patients.

The article "Survival analysis of comprehensive treatment in Chinese patients with metastatic melanoma: A retrospective analysis" was published in 2024. Journal: Skin Res Technol.

Each subgroup analysis also suggested that patients could benefit from immunotherapy regardless of age, BRAF V600E status, LDH, bone metastasis, and chemotherapy (Figure 2)

**FIGURE 2:** Forest plot: subgroup analysis suggested that the prognosis factors affecting OS were performed in univariate analysis, and each subgroup could benefit from immunotherapy. OS, overall survival.

## 4 DISCUSSION

The pathological types and biological characteristics of melanoma in China are different from those in western countries. The patients in China are mainly acral and mucosa types (about 41.8% and 22.6%), while the skin melanoma are dominant in western countries (about 90%).^3^, ^4^, ^5^ Immune checkpoint inhibitors have become the standard treatment regimen for advanced or metastatic cutaneous melanoma, however, there are limited data on acral and mucosal melanoma receiving immune checkpoint inhibitors, and they respond poorly to immunotherapy compared to the skin.^8^, ^13^ A retrospective study, even in skin subtypes, anti‐PD‐1 mAbs were significantly less effective in Asians than in Caucasian.^14^ How to improve the prognosis of Asian patients with malignant melanoma is an urgent problem for us to solve.

This study included patients with acro and mucosal malignant melanoma, 26 acromalignant melanoma (49.1% of the total) and 17 mucosal malignant melanoma (32.1% of the total). The PD‐1 mAb was well tolerated by the treated patients, with a median PFS of 7 months and a median OS of 24 months. These data support that PD‐1 mAb can improve survival in Chinese patients with advanced or metastatic melanoma. However, the multivariate analysis results of this study also suggested that immunotherapy is a protective factor for OS, which also confirmed this view. It is worth mentioning that immune combination therapy accounted for 81.4% in this study, including combination chemotherapy and targeted drug therapy. Chemotherapy and antiangiogenesis‐targeted therapy may promote the response to immunotherapy.

Chemotherapy has been the main treatment of advanced malignant melanoma, including dacarbazine, temozolomide, albumin‐bound paclitaxel, and so forth. Dacarbazine was approved by the FDA as a standard chemotherapy regimen for melanoma treatment starting in 1975. Tmozolomide was similar to dacarbazine. A randomized phase III trial of temozolomide and dacarbazine in patients with metastatic melanoma showed that median OS was comparable (7.7 months for temozolomide and 6.4 months for dacarbazine, *p* = 0.20) and similar response rates between them (temozolomide was

13.5%, dacarbazine was 12.1%).^15^ A phase III randomized controlled clinical trial of albumin‐bound paclitaxel and dacarbazine in first‐line treatment of metastatic melanoma suggested a median PFS of 4.8 months for albumin‐bound paclitaxel, 2.5 months (*p* = 0.044), median OS of 12.6 months for albumin‐bound paclitaxel, 10.5 months (*p* = 0.271), and overall remission rates of albumin‐bound paclitaxine, 15% and 11% (*p* = 0.239).^16^ These results suggest that chemotherapy has some activity on the treatment of advanced malignant melanoma but has limited impact on survival. The median OS of patients receiving chemotherapy in this study was significantly shorter compared to patients not receiving chemotherapy (14 months vs. 35 months, *p* = 0, Table 9), and the univariate analysis also suggested that chemotherapy was one of the adverse prognosis factors for OS (*p* < 0.1, Table 7). No conversion survival benefit from chemotherapy may be related to its chemotherapy toxicity, including myelosuppression, nausea and vomiting, increased toxic and side effects, decreased quality of life, and no improvement in OS rate.

The article "Survival analysis of comprehensive treatment in Chinese patients with metastatic melanoma: A retrospective analysis" was published in 2024. Journal: Skin Res Technol.

**TABLE 9:** Overall survival comparison between patients with or without chemo (date from first line to date of events).

	Median	95% CI	*p*‐value
Chemo	14.0	5.816–22.184	0.024
No chemo	35.0	33.704–36.296	
Total	19.0	10.035–27.965	

It is worth mentioning that, although there is no head‐to‐head clinical study on immunity and chemotherapy, previous studies suggest that chemotherapy can produce immunomodulatory effects, which may produce synergistic effects with immunotherapy through the destruction of immunosuppression pathway, the enhancement of cytotoxic T cell response, and the effect on tumor immune microenvironment.^17^, ^18^ In this study, 18 patients had combined immunotherapy or sequential chemotherapy (41.9% of the total population), which may be responsible for the longer OS than previous reports.

In this study, there were 17 immune combination targeted therapy (39.5% of the total population). Although targeted therapy was not a protective factor for OS in multivariate analysis, immune combination targeted therapy may be one of the reasons for prolonged OS of immune checkpoint inhibitors. This study had a limited number of samples and aimed to analyze the effect of immunotherapy on metastatic malignant black survival, and did not separately analyze BRAF and MEK inhibitors with anti‐angiogenic targeted therapy. Malignant melanoma with BRAF‐V600 mutation, either targeted therapy after immunotherapy as recommended by NCCN guidelines, or immunization before targeted^19^ as recommended by DREAMseq studies, suggests that BRAF‐V600 mutant metastatic melanoma could benefit from immunotherapy. The subgroup analysis of this study also suggested that it could benefit from immunotherapy regardless of the presence of mutations in BRAF‐V600E. Antiangiogenic, targeted therapy can also reverse the immunosuppressive tumor microenvironment by normalizing blood vessels, and subsequently induce T cell infiltration and activation, thereby promoting immunotherapy‐active.^20^

The article "Survival analysis of comprehensive treatment in Chinese patients with metastatic melanoma: A retrospective analysis" was published in 2024. Journal: Skin Res Technol.

This study also found that combined topical therapy showed a trend of survival benefit from no local treatment, with PD‐1 arterial perfusion therapy (16 patients, 30%). A study of PD‐1 in our department from January 2019 in 11 patients with advanced acral or mucosal melanoma through August 2020 with a median follow‐up of 8 months. The results showed that the response rate (RR) and disease control rate (DCR) of patients (7 acral melanoma, 4 mucosal melanoma) were 54.5% and 90.9%, respectively, no grade 3–4 adverse events or major complications were observed during the study period, and the median PFS was 10 months.^21^ Combined local therapy facilitates rapid tumor control, and combined immunotherapy facilitates prolonged survival.

We must admit that there are some limitations to our study. This was a retrospective study, which may cause some selection bias, in addition, we selected patients undergoing medication throughout in our department with a relatively small sample size. But our cohort also included some patients with poor medical condition and was more representative of the actual clinical situation.

In conclusion, immune checkpoint inhibitors can improve the prognosis of Chinese patients with malignant melanoma, and combination therapy will be a trend to improve the immune response and prolong survival, but which combination strategy will be the preferred regimen for Chinese patients with malignant melanoma still needs to be determined in more randomized clinical trials. More exploratory studies and establishing comprehensive treatment strategies are needed to improve the prognosis of Chinese melanoma patients.

## AUTHOR CONTRIBUTIONS

Qianqi Chen carried out the conception and design of this study. Acquisition of data was conducted by Yan Zhao and Pupu Li. Jiangman Duan, Xiaohong Fu, Yueqiang Tang, and Yinan Ma conducted the Statistical analysis, data interpretation and drafted the manuscript along with Qianqi Chen, that was later revised by all the authors. The funding was obtained by Qiming Zhou and supervised the whole study. All the authors approved the final version of the manuscript.

The article "Survival analysis of comprehensive treatment in Chinese patients with metastatic melanoma: A retrospective analysis" was published in 2024. Journal: Skin Res Technol.

## CONFLICT OF INTEREST STATEMENT

The authors declared that they have no conflicts of interest regarding this work.

## ETHICAL APPROVAL AND CONSENT TO PARTICIPATE

This research was approved by Ethic Review Board of Huazhong University of Science and Technology Union Shenzhen Hospital, Nanshan 518000, Shenzhen, Guangdong Province, PR China. All the necessary formalities for the informed consent of the patients were fulfilled according to the local regulation and Declaration of Helsinki.

## PATIENT CONSENT FOR PUBLICATION

All the patients involved in this study provided written informed consent for the publication of any data and/or accompanying images.

## Data Availability

The data that support the findings of this study are available from the corresponding author upon reasonable request.
